# Cognitive Dysfunction of Pregnant Women with Gestational Diabetes Mellitus in Perinatal Period

**DOI:** 10.1155/2021/2302379

**Published:** 2021-08-06

**Authors:** Siriguleng Sana, Xijin Deng, Lei Guo, Xunhong Wang, Enyou Li

**Affiliations:** ^1^Department of Anesthesiology, The First Affiliated Hospital of Harbin Medical University, Harbin 150001, Heilongjiang Province, China; ^2^Department of Anesthesiology, The Second Affiliated Hospital of Harbin Medical University, Harbin 150001, Heilongjiang Province, China; ^3^Department of Obstetrics, The First Affiliated Hospital of Harbin Medical University, Harbin 150001, Heilongjiang Province, China

## Abstract

**Purpose:**

To explore whether pregnant women with gestational diabetes mellitus (GDM) had cognitive impairment and assess cognitive function in normal pregnant women.

**Methods:**

A total of 75 consecutive women diagnosed with GDM (GDM group), 70 normal pregnant women (NP group) without diabetes and matched for age, and 51 female volunteers (CG group) with the similar age level, normal blood glucose, and nonpregnancy were included in the study. For the assessment of cognitive functions, Montreal Cognitive Assessment (MoCA) was performed. Venous blood samples were collected to measure blood glucose, glycated hemoglobin (HbA1c), methylglyoxal (MGO), beta amyloid (A*β*), and tau protein.

**Results:**

The score of MoCA of GDM was lowest, and the score of the NP group was lower than volunteers (*P* < 0.05). The incidence of cognitive dysfunction increased significantly in the GDM group with statistical significance (*P* < 0.05). The levels of tau and MGO in the GDM group were significantly less than those in the NP and CG groups, and A*β* in the GDM group was significantly more than that in the NP and CG groups (*P* < 0.05), but the differences between NP and CG groups were not statistically significant (*P* < 0.05).

**Conclusion:**

The pregnant women with GDM showed a significant decline in cognitive function, and the normal pregnant women also showed a decline in cognitive function which is very light.

## 1. Introduction

Gestational diabetes mellitus (GDM) occurs in pregnant women who were not diagnosed with diabetes before pregnancy but have abnormal result of OGTT or/and high blood glucose levels during pregnancy, usually around the 24th week, by the American Diabetes Association [1]. According to the most recent International Diabetes Federation (IDF) estimates (2019), GDM affects approximately 13.2% of pregnancies worldwide, representing approximately 17 million births annually. The risk factors of GDM include older age, overweight and obesity, previous GDM, a family history of diabetes, and a history of stillbirth or giving birth to an infant with a congenital abnormality. GDM usually exists as a transient disorder during pregnancy and resolves once the pregnancy ends. However, it can have long-lasting health consequences, including increased risk for type 2 diabetes (T2DM) and cardiovascular disease (CVD) in the mother, and future obesity, and/or GDM in the child [2].

The pathogenesis of GDM is still not clear, although there are many risk factors, similar to type 2 diabetes (T2DM). Cognitive dysfunction in cases with long standing T2DM has been widely reported [3]. And, decline of verbal memory, associate learning, and verbal recall in normal pregnant women have been reported [4–6]. However, few studies have identified cognitive dysfunction in GDM patients [7]. Therefore, this study observed the cognitive function of pregnant women, especially who are suffering from GDM and tried to improve the evidence from the serological point of view.

## 2. Materials and Methods

### 2.1. Subjects and Protocol

Patients aged 18–35 years with American Society of Anaesthesiologists (ASA) physical status I-II were admitted to the study. A total of 101 consecutive women with GDM who were diagnosed, followed, and treated at the First Affiliated Hospital of Harbin Medical University included in the study. 76 pregnant women without diabetes and matched for age constituted the normal pregnancy group (NP). And, we recruited 51 female volunteers with the similar age level, normal blood glucose, and are not pregnant formed the control group (CG). All the patients and volunteers read and signed the informed consent forms before enrolling in the study. The study protocol was approved by the Ethics Committee of First Affiliated Hospital of Harbin Medical University, which was registered with the Chinese Clinical Trial Register (registration number: ChiCTR2000038703).

GDM was diagnosed with at least one abnormal result during OGTT: plasma glucose during fasting ≥92 mg/dL (5.1 mmol/L) or at 1 h ≥180 mg/dL (10.0 mmol/L) or at 2 h ≥153 mg/dL (8.5 mmol/L). Cases with fasting plasma glucose ≥126 mg/dL (7.0 mmol/L), HbA1c ≥6.5%, or a random plasma glucose ≥200 mg/dL (11.1 mmol/L) were diagnosed with overt diabetes and excluded. Cases with pregestational T1 or T2DM were not included in the study. Cases with unnatural pregnancy or gestational period <37 weeks or >41 weeks were excluded. Subjects on medications affecting cognitive functions including corticosteroids, antidepressants, or antiepileptics were also not included. Additionally, subjects suffering from any chronic metabolic, endocrine, inflammatory diseases, cancer, subjects who had drug or alcohol dependency, history of major brain abnormalities (e.g., tumors and hydrocephaly), epilepsy, and Parkinson's disease were excluded. The Hamilton Depression Rating Scale (HAMD) was used to assess the psychological status of pregnant women and those with a score of more than 7 might have depression and were excluded [8].

On the survey date, all enrolled patients underwent routine medical history inquiries, physical examinations, and laboratory measurements. Clinical research coordinators used a standard questionnaire to collect information on demographic characteristics and a medical history. There were no racial/ethnic, educational, or socioeconomic differences between the groups (Table 1). All pregnant women were instructed to maintain their usual physical activity and diet for at least 3 days before the survey. After an overnight fasting of ≥10 h, venous blood samples were collected to measure blood lipids, glycated hemoglobin (HbA1c), methylglyoxal (MGO), beta amyloid (A*β*), and tau protein activity. Blood samples were stored at −80°C, and all parameters were measured within 6 months of sample collection.

### 2.2. Assessment of Cognitive Function

For the assessment of cognitive functions, Montreal Cognitive Assessment (MoCA), which is a brief cognitive screen across a variety of clinical settings and widely used, was performed [9]. The assessment was conducted in a quiet room without distractions by a physical therapist trained in the administration of the MoCA questionnaire. The total score of the respondents with less than 12 years of education can be increased by one point on the premise that the total score does not exceed 30 points.

### 2.3. Statistical Analysis

The data were statistically analyzed with the SPSS 19.0 package program. All measures were tested for normality and homogeneity of variance. Normally distributed data are expressed as means ± SD. Continuous variables with normal distribution were compared by using the Student's *t*-test and those with nonnormal distributions were compared by using the Mann–Whitney *U*-test, and the multiple comparison between groups was performed by the LSD method. The count data were described by percentage, and the comparison between groups was performed by *χ*^2^-test, which were two-sided tests. *P* < 0.05 was considered statistically significant.

## 3. Results

The study plan included 177 pregnant women and 51 volunteers, and a total of 145 pregnant women and 51 volunteers were eventually enrolled, including 75 pregnant women with GDM in the GDM group, 70 normal pregnant women in the NP group, and 51 volunteers in the CG group (Figure 1).

Compared with the CG group, the score of visuospatial/executive, attention, delayed recall, and total was significantly lower in the GDM and NP group, and the language score was lower in the GDM group (*P* < 0.05). Compared with the NP group, the score of visuospatial/executive, language, delayed recall, and total was significantly lower in the GDM group (*P* < 0.05) (Table 2).

The levels of tau and MGO in the GDM group was significantly less than these in the NP and CG groups (*P* < 0.05), but the differences between NP and CG groups were not statistically significant (*P* < 0.05). The level of A*β* in the GDM group was significantly more than that in the NP and CG groups (*P* < 0.05), and the differences between NP and CG groups were not statistically significant (*P* < 0.05), though the level of tau in NP was more than that in the CG group (Figure 2).

## 4. Discussion

The viewpoint that pregnant women suffer from deficits in memory is widespread, while the related documents are limited, especially in humans [10]. In this study, we found pregnant women did have a decrease in cognitive function scores. And, the incidence of cognitive dysfunction in pregnant women with GDM is much higher than that in normal pregnant women. Among all the tests of MoCA score, the most significant change was delayed recall.

In fact, the effect of childbirth on women's cognitive ability is an obscure issue, because it may affect the job opportunities of working women of childbearing age. So, we discuss the impact of pregnancy on women's cognitive function with caution. Actually, the average score of normal pregnant women is indeed lower than that of volunteer women with the similar age, from the MoCA score point of view. But the degree of this cognitive function decline is lighter comparing with the pregnant women with GDM. In the late stages of pregnancy, most pregnant women will be out of the working environment, and the brain belongs to excessive relaxation state in terms of cognition that may be one of the reasons of the mild cognitive decline in pregnant women [11, 12]. Mild stress, anxiety, and depression about childbirth during pregnancy may also affect the cognitive function of pregnant women to a certain extent [13, 14]. However, most of these bad emotions during pregnancy would disappear with childbirth. On the other hand, the levels of A*β* and tau were much closer to normal women. Therefore, we think the decline of cognitive of pregnant women was minimal and less influential.

However, cognitive decline in women with GDM is less optimistic. At first, the average score of MoCA was the lowest, and the difference was statistically significant. And, the levels of tau were lowest, while those of A*β* were highest. The changes of these plasma markers should be paid much more attention, though the pregnant women with GDM may need to face more serious emotions problems that may affect cognitive function.

A*β* and tau are a group of plasma markers related to cognitive function. The primary pathological changes in Alzheimer's disease (AD) are intracellular neurofibrillary tangles induced by tau phosphorylation and intercellular senile plaque accumulation induced by oligomerization of A*β* protein [15]. The toxic effects of A*β* can lead to dysfunction in neurotrophic factor expression. Compared with cognitive impairment, we are more worried about the changes of serum markers, suggesting that the effect of this cognitive impairment is long-term and even can cause AD.

MGO is advanced glycation endproducts (AGEs), a highly reactive *α*-dicarbonyl that is mainly generated as a byproduct of glycolysis and auto-oxidation of glucose which can initiate potentially deleterious changes, leading to protein dysfunction, have raised concern in relation to healthy living [16, 17]. MGO has been implicated in the pathogenesis of T2DM, vascular complications of diabetes, and several other age-related chronic inflammatory diseases such as cardiovascular disease, cancer, and disorders of the central nervous system [18].

Increased levels of AGEs were reported in brains of AD patients and were also found to be associated with the amyloid plaques and the neurofibrillary tangles (NFTs) [19, 20]. Many studies have reported the capacity of MGO intermediates to induce cellular damage and contribute to the pathogenesis of many neurodegenerative diseases [21]. For instance, increased intracellular reactive oxygen species production, tau hyperphosphorylation, and mitochondrial dysfunction were observed in neuronal cells following MGO treatment [22]. The intracerebroventricular (ICV) administration of MGO induced tau hyperphosphorylation and caused hippocampal damage and memory impairment in mice [23]. So, we believe that the increasing MGO of GDM pregnant women is the reason of mild cognition decline.

In this experiment, the results of MOCA score and serum indicators of perinatal GDM pregnant women are consistent. The mechanism of memory loss in pregnant women with perinatal GDM may be complex. In recent years, more and more attention has been paid to the relationship between diabetes and cognitive impairment. Compared with the general population, cognitive dysfunction in patients with type 2 diabetes is 1.5–2 times higher [24, 25]. Many studies support this view, and diabetic patients have a greater risk of cognitive impairment [26, 27]. The mechanism may be related to protein aggregation, insulin damage, oxidative stress, inflammatory reaction, and the generation of diabetes end products. This study is also in line with this view.

GDM is considered to be a prediabetic state, and the pathology of them is significantly correlated. In recent years, studies have shown that abnormal lipid metabolism can be widely involved in the pathophysiological process of a series of metabolic diseases such as obesity and type 2 diabetes by mediating oxidative stress and other signal transduction pathways. There are many studies on oxidative stress and inflammatory reaction in GDM pregnant women. Monitoring the serum C-reactive protein (CRP) level in early pregnancy is of great significance for predicting GDM [28]. Moreover, the study indicates that interleukin-6 (IL-6) and 8-isoprostaglandin F2 *α* (8-iso-pgf2 *α*) are significantly increased in GDM. These mechanisms may be involved in the cognitive dysfunction of GDM pregnant women, and the specific mechanism needs to be further studied.

## 5. Conclusion

The pregnant women with GDM have a significant decline in cognitive function, and the normal pregnant women have also a decline in cognitive function which very light.

## Figures and Tables

**Figure 1:** Patient recruitment flowchart.

**Figure 2:** Concentration of (a) A*β*-42, (b) tau, and (c) MGO of each group; compared with NP group, ^#^*P* < 0.05; compared with CG group, ^*∗*^*P* < 0.05.

**Table 1:** Demographic characteristics.

	GDM	NP	CG	F	*P*
Sample	73	70	51		
Age	29.70 ± 3.06	29.56 ± 3.39	29.52 ± 3.33	0.06	0.95
Height (cm)	164.75 ± 4.58	164.61 ± 5.08	164.28 ± 5.03	0.14	0.87
Weight (kg)	77.86 ± 10.46	74.25 ± 8.97	58.65 ± 7.49	68.32	<0.001
Glucose	4.95 ± 1.29	3.99 ± 0.76	4.69 ± 0.55	18.90	<0.001
Hba1c (%)	5.83 ± 0.63	4.74 ± 0.93		8.24	<0.001
Education (%)				0.02	0.99
Primary school	4 (5.5)	3 (4.3)	1 (2.0)		
High school	19 (26.0)	18 (25.7)	14 (27.5)		
University	50 (68.5)	49 (70.0)	36 (70.6)		

Data are expressed as means ± SD or number.

**Table 2:** MoCA test score.

	GDM	NP	CG	*P* (GDM vs. NP)	*P* (GDM vs. CG)	*P* (NP vs. CG)
Sample	73	70	51			
Visuospatial/executive	4.42 ± 0.84	4.55 ± 0.63	4.94 ± 0.35	0.24	<0.001	0.002
Naming	3.00 ± 0.00	3.00 ± 0.00	3.00 ± 0.00	—	—	—
Attention	5.52 ± 0.84	5.57 ± 0.70	5.82 ± 0.27	0.66	0.02	0.04
Language	2.64 ± 0.52	2.82 ± 0.41	2.95 ± 0.21	0.01	<0.001	0.09
Abstraction	1.97 ± 0.15	1.97 ± 0.14	2.00 ± 0.00	—	—	—
Orientation	6.00 ± 0.00	5.99 ± 0.10	6.00 ± 0.00	—	—	—
Delayed recall	2.81 ± 1.15	3.62 ± 1.21	4.18 ± 0.91	<0.001	<0.001	0.01
Total	26.98 ± 1.79	28.01 ± 1.85	29.00 ± 1.18	<0.001	<0.001	<0.001

Data are expressed as means ± SD or number.

## Data Availability

The datasets generated during and/or analyzed during the current study are not publicly available but are available from the corresponding author on reasonable request.

## References

[1] American Diabetes Association (2016). Classification and diagnosis of diabetes. *Diabetes Care*.

[2] Plows J., Stanley J., Baker P., Reynolds C., Vickers M. (2018). The pathophysiology of gestational diabetes mellitus. *International Journal of Molecular Sciences*.

[3] Umegaki H., Hayashi T., Nomura H. (2013). Cognitive dysfunction: an emerging concept of a new diabetic complication in the elderly. *Geriatrics and Gerontology International*.

[4] Glynn L. M. (2010). Giving birth to a new brain: hormone exposures of pregnancy influence human memory. *Psychoneuroendocrinology*.

[5] Janes C., Casey P., Huntsdale C., Angus G. (1999). Memory in pregnancy. I: subjective experiences and objective assessment of implicit, explicit and working memory in primigravid and primiparous women. *Journal of Psychosomatic Obstetrics and Gynaecology*.

[6] Casey P., Huntsdale C., Angus G., Janes C. (1999). Memory in pregnancy. II: implicit, incidental, explicit, semantic, short-term, working and prospective memory in primigravid, multigravid and postpartum women. *Journal of Psychosomatic Obstetrics and Gynaecology*.

[7] Keskin F. E., Ozyazar M., Pala A. S. (2015). Evaluation of cognitive functions in gestational diabetes mellitus. *Experimental and Clinical Endocrinology & Diabetes*.

[8] Zimmerman M., Martinez J. H., Young D., Chelminski I., Dalrymple K. (2013). Severity classification on the Hamilton depression rating scale. *Journal of Affective Disorders*.

[9] O’Driscoll C., Shaikh M. (2017). Cross-cultural applicability of the montreal cognitive assessment (MoCA): a systematic review. *Journal of Alzheimer’s Disease*.

[10] Brown E., Schaffir J. (2019). Pregnancy brain: a review of cognitive changes in pregnancy and postpartum. *Obstetrical & gynecological survey*.

[11] Al-Thaqib A., Al-Sultan F., Al-Zahrani A. (2018). Brain training games enhance cognitive function in healthy subjects. *Medical science monitor basic research*.

[12] Nouchi R., Taki Y., Takeuchi H. (2013). Brain training game boosts executive functions, working memory and processing speed in the young adults: a randomized controlled trial. *PloS One*.

[13] Gawali N. B., Bulani V. D., Gursahani M. S., Deshpande P. S., Kothavade P. S., Juvekar A. R. (2017). Agmatine attenuates chronic unpredictable mild stress-induced anxiety, depression-like behaviours and cognitive impairment by modulating nitrergic signalling pathway. *Brain Research*.

[14] Glover V. (2014). Maternal depression, anxiety and stress during pregnancy and child outcome; what needs to be done. *Best Practice & Research Clinical Obstetrics&gynaecology*.

[15] Chen Q., Ma H., Guo X., Liu J., Gui T., Gai Z. (2019). Farnesoid X receptor (FXR) aggravates amyloid-*β*-triggered apoptosis by modulating the cAMP-response element-binding protein (CREB)/brain-derived neurotrophic factor (BDNF) pathway in vitro. *Medical Science Monitor : International Medical Journal of Experimental and Clinical Research*.

[16] Maessen D. E., Stehouwer C. D., Schalkwijk C. G. (2015). The role of methylglyoxal and the glyoxalase system in diabetes and other age-related diseases. *Clinical science (London, England : 1979)*.

[17] Wang Y., Hall L. M., Kujawa M. (2019). Methylglyoxal triggers human aortic endothelial cell dysfunction via modulation of the K (ATP)/MAPK pathway. *American Journal of Physiology Cell Physiology*.

[18] Schalkwijk C. G., Stehouwer C. D. A. (2020). Methylglyoxal, a highly reactive dicarbonyl compound, in diabetes, its vascular complications, and other age-related diseases. *Physiological Reviews*.

[19] Haddad M., Perrotte M., Khedher M. R. B. (2019). Methylglyoxal and glyoxal as potential peripheral markers for mci diagnosis and their effects on the expression of neurotrophic, inflammatory and neurodegenerative factors in neurons and in neuronal derived-extracellular vesicles. *International Journal of Molecular Sciences*.

[20] Lüth H. J., Ogunlade V., Kuhla B. (2005). Age- and stage-dependent accumulation of advanced glycation end products in intracellular deposits in normal and Alzheimer’s disease brains. *Cerebral Cortex (New York, NY : 1991)*.

[21] Li X. H., Xie J. Z., Jiang X. (2012). Methylglyoxal induces tau hyperphosphorylation via promoting AGEs formation. *NeuroMolecular Medicine*.

[22] Tajes M., Eraso-Pichot A., Rubio-Moscardó F. (2014). Methylglyoxal reduces mitochondrial potential and activates bax and caspase-3 in neurons: implications for Alzheimer’s disease. *Neuroscience Letters*.

[23] Chen Y. J., Huang X. B., Li Z. X., Yin L. L., Chen W. Q., Li L. (2010). Tenuigenin protects cultured hippocampal neurons against methylglyoxal-induced neurotoxicity. *European Journal of Pharmacology*.

[24] Luchsinger J. A., Reitz C., Patel B., Tang M. X., Manly J. J., Mayeux R. (2007). Relation of diabetes to mild cognitive impairment. *Archives of Neurology*.

[25] Reijmer Y. D., van den Berg E., Ruis C., Kappelle L. J., Biessels G. J. (2010). Cognitive dysfunction in patients with type 2 diabetes. *Diabetes/metabolism research and reviews*.

[26] Feinkohl I., Winterer G., Pischon T. (2017). Diabetes is associated with risk of postoperative cognitive dysfunction: a meta-analysis. *Diabetes/metabolism research and reviews*.

[27] Zhang X., Dong H., Zhang S., Lu S., Sun J., Qian Y. (2015). Enhancement of LPS-induced microglial inflammation response via TLR4 under high glucose conditions. *Cellular Physiology and Biochemistry: International Journal of Experimental Cellular Physiology, Biochemistry, and Pharmacology*.

[28] Fatema N., Deeba F., Akter S. (2016). CRP (C-reactive protein) in early pregnancy predictor for development of GDM. *Mymensingh Medical Journal : MMJ*.

